# Investigation of FGFR2-IIIC Signaling via FGF-2 Ligand for Advancing GCT Stromal Cell Differentiation

This article has been retracted.

**DOI:** 10.1371/journal.pone.0046769

**Published:** 2012-10-11

**Authors:** Shalini Singh, Mohini Singh, Isabella W. Y. Mak, Robert Turcotte, Michelle Ghert

**Affiliations:** 1 Department of Surgery, McMaster University, Hamilton, Ontario, Canada; 2 Department of Orthopaedic Surgery, McGill University Health Centre, Montreal General Hospital, Quebec, Canada; Faculté de médecine de Nantes, France

## Abstract

Giant cell tumor of bone (GCT) is an aggressive bone tumor consisting of multinucleated osteoclast-like giant cells and proliferating osteoblast-like stromal cells. The signaling mechanism involved in GCT stromal cell osteoblastic differentiation is not fully understood. Previous work in our lab reported that GCT stromal cells express high levels of TWIST1, a master transcription factor in skeletal development, which in turn down-regulates Runx2 expression and prevents terminal osteoblastic differentiation in these cells. The purpose of this study was to determine the upstream regulation of TWIST1 in GCT cells. Using GCT stromal cells obtained from patient specimens, we demonstrated that fibroblast growth factor receptor (FGFR)-2 signaling plays an essential role in bone development and promotes differentiation of immature osteoblastic cells. Fibroblast growth factor (FGF)-2 stimulates FGFR-2 expression, resulting in decreased TWIST1 expression and increased Runx2, alkaline phosphastase (ALP) and osteopontin (OPN) expression. Inhibition of FGFR-2 through siRNA decreased the expression of ALP, Runx2 and OPN in GCT stromal cells. Our study also confirmed that FGF-2 ligand activates downstream ERK1/2 signaling and pharmacological inhibition of the ERK1/2 signaling pathway suppresses FGF-2 stimulated osteogenic differentiation in these cells. Our results indicate a significant role of FGFR-2 signaling in osteoblastic differentiation in GCT stromal cells.

## Introduction

Giant cell tumor of bone (GCT) is an aggressive osteolytic and potentially metastatic bone tumor. GCT typically prompts the formation of a local osteolytic lesion at the epiphyseal regions of the long bones such as the distal femur, the proximal tibia, and the distal radius [1]. High recurrence rates of 18–60% following aggressive surgical resection have been reported for GCT, which occasionally undergoes malignant transformation [2]–[5]. Cell culture experiments have shown that the preosteoblast-like GCT mesenchymal stromal cells are the only proliferating component of GCT, and are arrested in an immature differentiation state [6], [7].

The formation of skeletal elements is controlled by a complex network of signaling molecules that regulate the differentiation of mesenchymal stromal cells into osteoblasts and terminal differentiation into osteocytes under appropriate stimulation by hormones and local factors such as fibroblast growth factors (FGFs) [8]–[10]. FGF signaling plays an essential role in bone development, promoting proliferation of immature osteoblast/osteoprogenitor cells and increasing apoptosis upon exposure of cells to differentiation media [11], [12]. Four fibroblast growth factor receptor genes (FGFR1–4) have been identified in mammalian developmental processes.

The specificity of FGFR1–4 is regulated in a tissue specific manner. FGFR-1 acts as a transducer of FGF signals in osteoblast proliferation [13]. In contrast FGFR-2 has been shown to enhance osteoblast differentiation in mesenchymal stem cells [14], [15] whereas FGFR3 and 4 are generally restricted to chondrocytes [16], [17]. Splice variants of the FGFR-2 gene are classified by their ability to bind specific ligands [18]. FGF receptor 2-IIIc (FGFR2-IIIc) has the ability to bind both FGF-1 and FGF-2 with a high affinity due to its possession of the IIIc exon [9], [18]–[21].

The FGFRs are tyrosine kinases which possess three extracellular immunoglobulin-like domains, a trans-membrane region and a cytoplasmic split tyrosine kinase domain which is activated upon FGF binding [22]. FGF binding to FGFR leads auto phosphorylation of intracellular tyrosine residues. FGFR phosphorylation facilitates the recruitment of numerous signaling proteins [23] which subsequently activates various signaling pathways downstream of FGFR, including the extracellular-signal-regulated kinase 1/2 (ERK1/2) pathway. ERK1/2 is one of the main downstream targets of activated FGFRs. In the bone environment, activation of ERK1/2 has been found to enhance osteoblast gene expression [24].

The transcription factor TWIST1 also plays an important role in bone and cranial suture development, and is expressed in skeletal mesenchymal cells, primary osteoblastic and preosteoblasts cells. Runx2 is a master osteogenic regulator and acts as an inducer and regulator of osteoblast differentiation in the osteoblast lineage [25]–[28]. We have previously observed a high expression of TWIST1 in GCT stromal cells [29]. TWIST1 is an upstream regulator of Runx2 that acts to downregulate Runx2 expression, prevent terminal osteoblastic differentiation, and plays an important role in specifically disrupting the balance in bone formation and resorption in GCT [29].

However, the mechanism through which TWIST1 regulates GCT stromal cell differentiation remains unclear. Based on our previous work, we hypothesized that FGF-2 ligand signaling through FGFR2-IIIc receptor suppresses TWIST1 expression and may have a positive effect on the commitment and differentiation of osteoblast precursor cells. In this study, our main focus was to investigate the FGFR2-IIIC signaling via FGF-2 ligand for GCT stromal cells differentiation. We have investigated the effect of FGF-2 signaling on GCT cells in osteogenic differentiation and determined the mechanisms involved in the regulation of osteoblast commitment and differentiation. We have also studied the role of FGFR2-IIIc in the regulation of the TWIST1 and Runx2 osteoblastic transcription factors and its activation of the ERK1/2 signaling in GCT stromal cells.

## Materials and Methods

### Ethics Statement

We established primary cell cultures of GCT stromal cells from fresh GCT tissue obtained from four patients following the Hamilton Health Sciences and McMaster University Ethics Board approval and written patient consent.

### Primary cell culture and FGF-2 treatment

The tissue was processed and maintained in DMEM containing 10% FBS, 2 mM glutamine and 100 U/mL streptomycin antibiotics. The resulting cell suspension together with macerated tissue was cultured in 37°C humidified air with 5% CO_2_. Following several successive passages, the mesenchymal stromal cells became the homogeneous cell type whereas the multinucleated giant cells were eliminated from culture. Primary cultures of the proliferating homogenous stromal tumor cell population obtained after the fifth or sixth passage (without any hematopoietic markers) and up to the tenth passage were used for experiments [30], [31]. GCT-stromal cells were incubated in media containing 50 nmol/L ascorbic acid, 3 mM inorganic phosphate (NaH_2_PO_4_) and a range of dilution from 10 to 40 ng/ml of FGF-2 (Minneapolis, MN). Human fetal osteoblast (hFOB) 1.19 cells (American Type Culture Collection, ATCC# CRL- 11372) were used as a control cell line to compare the endogenous FGFR-2IIIc expression in GCT stromal cells. The hFOB cell line is a clonal, conditionally immortalized human fetal cell line capable of osteoblastic differentiation and bone formation.

### Plasmid construction

A TWIST1 open-reading frame was amplified by PCR from the plasmid purchased from Origene (Rockville, MD) using oligonucleotides cgcggatccgcgatgatgcaggacgtgtcc and ccggaattccggctagtgggacgcgacat, containing *BamHI* and *EcoRI* restriction sites, respectively. After *BamHI* and *EcoRI* digestion, the open-reading frame was ligated into a pcDNA3.1 vector and confirmed by sequencing. GCT cells were transfected using an electroporation method [29]. After 48-h post-transfection, cells were harvested for RNA isolation.

### RNA Isolation and RT-PCR

Total RNA extraction was performed by TRIZOL Reagent (Sigma) according to the manufacturer's protocol. The resuspended RNA samples were treated with ribonuclease A (RNase A)-free DNaseI for 1 h at 37°C to remove residual genomic DNA. One microgram of total RNA was incubated with 2 ml primer cocktail at 68°C and subjected to reverse transcription (RT) using Superscript III reverse transcriptase (Invitrogen) for cDNA synthesis. PCR was carried out using Prime Taq Premix and reactions were carried out in the PCR thermal cycler (Applied Biosystems, Foster City, CA, USA). Expression of the ribosomal protein 18 (RPS18) was used as internal control. Primer sequences are listed in **Table 1**.

**Table 1:** Primers sequences designed for real time RT-polymerase chain (PCR) reaction.

Gene symbol	Oligonucletides
ALP	CATTGGCACCTGCCTTACTA
	ACGTTGGTGTTGAGCTTCTG
RunX2	TCTGGCCTTCCACTCTCAGT
	AAGGTGGCTGGATAGTGCAT
TWIST	TACATCGACTTCCTCTACCAGGTC
	TAGTGGGACGCGGACATGGA
OPN	AGTTTCGCAGACCTGACATCCAGT
	TTCATAACTGTCCTTCCCACGGCT
RPS18	GATGGGCGGCGGAAAATAG
	GCGTGGATTCTGCATAATGGT

### Protein Extraction and Western blot analysis for TWIST1, Runx2 and Osteopontin

To detect protein expression, we isolated protein from FGF-2 treated and untreated GCT stromal cells. After 48 h of incubation, cells were lysed with NP-40 containing lysis buffer (10 mM Tris, pH 7.4, 10 mM NaCl, 5 mM MgCl2, 0.5% NP-40) to disrupt the cell membrane and the cell lysate was centrifuged at 500 g for 5 min at 4°C. The supernatant (cytoplasmic fraction) was removed. Proteins were denatured by boiling in sample buffer, separated on 12% SDS–PAGE, transferred onto a PVDF membrane (Immobilon TM-PSQ, Millipore), and blocked overnight in 5% non-fat powdered milk in TBST (10 mM Tris–HCl pH 7.5, 100 mM NaCl, 0.1% (v/v) Tween-20). Mouse monoclonal anti-TWIST1 antibody, mouse anti-Runx2 antibody, and mouse anti-osteopontin antibody, rabbit anti ERK1/2 and rabbit anti phosphorylated ERK1/2 (1∶1,000 diluted in TBST) (Abcam) were used for protein detection. Peroxidase conjugated goat anti-mouse, and anti-rabbit IgG (1∶5,000 diluted in TBST) (Promega) was used as a secondary antibody. Western blots were quantified with Image J program.

### Alizarin Red staining for bone nodule formation

Mineralization was assessed in FGF-2 treated GCT stromal cells on day 28 using an Alizarin Red-S staining assay. Cells were washed twice with PBS and fixed in 10% neutral buffered formalin (Fisher Scientific) for 30 min at room temperature. After washing with distilled water twice, cell were fixed and the matrix stained for 10 min with 0.02 g/mL Alizarin Red-S stain (pH 4.2) (Sigma-Aldrich) and visualized with an Olympus microscope to identify the presence or absence of bone nodule formation.

### ALP activity assay

The cells were washed with PBS and lysed with NP-40 containing lysis buffer (10 mM Tris, pH 7.4, 10 mM NaCl, 5 mM MgCl2, 0.5% NP-40) solution. ALP activity of the lysates was determined using p-nitrophenol-phosphate as a substrate. In brief, 50 µl of the cell lysate supernatant was mixed with 50 µl of the substrate solution (p-nitro-phenyl phosphate substrate solution diluted in ALP buffer for ALP measurement or p-nitro-phenyl phosphate substrate solution diluted in acid phosphatase buffer and incubated at 37°C for 30 min. Stop solution (50 µl, 0.9 N NaOH) was added to each well and the absorbance was measured at 405 nm with a spectrophotometer. Total protein content in aliquots of the same samples was determined using Bradford reagent (Sigma-Aldrich). The amount of ALP activity was divided by the amount of total protein for normalization.

### siRNA Transfection

Mesenchymal stromal cells of GCT were trypsinized and transfected with FGFR-2 small interfering RNAs (siRNAs) via electroporation. The cells were then washed and resuspended in Optimem reduce serum media (Gibco, Invitrogen, Canada). Subsequently, the cell suspension was mixed with 200 nM of FGFR-2 siRNA (Invitrogen), a positive Silencer™ siRNA control against GAPDH, or a non-specific negative control#1 (Ambion Inc.). Stromal cells with the siRNA mixture were electroporated using the Gene Pulser II electroporation apparatus (Bio-Rad laboratories) under a single-pulse protocol with optimized combination of voltage and capacitance. After 48 h of transfection, cells were harvested for RNA isolation. RPS18 was selected as housekeeping genes for normalization in real time PCR analysis.

### Immunofluorescence assay

Cells were grown on cover slips and were fixed with 4% paraformaldehyde for 20 min at room temperature (RT), and permeabilized with 0.2% Triton x-100 for 5 min. Subsequently, these slides were incubated for 1 h at RT with antibodies (anti-Osteopontin,). Slides were further incubated in secondary antibody (Texas red conjugated goat-anti rabbit and alexa 488 goat anti-mouse antibodies) for 1 h at RT. Slides were washed and incubated with DAPI for 3 min at RT and mounted with 50% glycerol and visualized with fluorescence microscopy.

### XTT cell proliferation assay

The XTT assay is based on the cleavage of the yellow tetrazolium salt XTT to form an orange formazan dye by metabolically active cells. We seeded 1000 cells with 100 µl of culture medium with FGF-2 and without FGF-2 in a 96 well plate, and after 48 h of culture the XTT assay was performed following the manufacturer's protocol (Roche Diagnostics). The absorbance was measured at 450 nm using a UV plate reader.

### Signaling pathway inhibition

The culture medium of the GCT stromal cells was replaced with serum-free medium containing ERK inhibitor 1 nM (R&D Systems). The effects of signaling pathway inhibitor kinase (ERK)-PD98059 with FGF-2 (20 ng/ml) were used. After 24 h of exposure to FGF-2 and inhibitor in GCT stromal cells the lysate were collected and analyzed. The expressions of TWIST1, ALP, OPN and OC were evaluated using real-time polymerase chain reaction (PCR).

### Statistical analysis

Statistical analyses for the real-time PCR were performed using the two sample independent student's t-test. The average value within each experiment was expressed relative to the expression of the internal control gene. *P*-value of <0.05 was considered statistically significant.

## Results

### Expression of FGF receptor 2-IIIc in GCT stromal cells

We determined the endogenous expression of FGFR2-IIIb and FGFR2-IIIc in GCT stromal cells obtained from four patient samples. FGFR2-IIIb and FGFR2-IIIc expression was analyzed with semi-quantitative RT-PCR using FGFR2-IIIb and FGFR2-IIIc specific primers. FGFR2-IIIb and FGFR2-IIIc endogenous expression was detected in all 4 GCT cell lines. Ribosomal protein S18 (RPS18) was used as an internal control (**Fig. 1a**). We further analyzed the expression of FGFR2-IIIb and FGFR2-IIIc by quantitative real-time RT-PCR. Interestingly, qRT-PCR analysis revealed significantly higher expression of FGFR2-IIIc in all GCT stromal cells when compared to hFOB 1.19 control cells using the two-sample independent student's *t*-test (*P*≤0.01) (**Fig. 1b**). Furthermore, we did not observe any quantitatively significant FGFR2-IIIb expression (data not shown). An increase was detected FGFR2-IIIc expression in response to FGF-2 ligand stimulation in GCT stromal cells (**Fig. 1c**). Therefore further experiments focused on FGFR2-IIIc signaling in GCT.

**Figure 1:** Semi-quantitative PCR. (**a**). Endogenous expression of FGFR2-IIIb and FGFR-2IIIc in GCT stromal cells using FGFR2 specific primers. (**b**). Real-time PCR of cDNA from GCT stromal cell lysates showing expression of FGFR2-IIIc relative to hFOB 1.19 cells (“hFOB”). Results are the average of three replicate experiments. (**c**). An increase in expression of FGFR-2IIIc is in response to FGF-2 ligand in GCT stromal cell in a dose dependent manner. Results are the average of three replicate experiments.

### FGF-2 effects on bone nodule formation and cell proliferation in GCT stromal cells

To investigate the role of FGF-2 signaling on osteoblastic proliferation and bone nodule formation, cells were treated with FGF-2 supplemented media for 4 weeks. We observed that FGF-2 treated cells promoted matrix mineralization and bone nodule formation in GCT cells when compared to untreated cells using alizarin and von kossa staining (**Fig. 2a, 2b**). To determine cell viability and proliferation, XTT assays were performed on GCT stromal cells with and without FGF-2 treatment. We observed decreased mitochondrial activity in GCT cells treated with an increasing FGF-2 dosage when compared to untreated GCT stromal cells after 48 h, indicating decreased proliferation and cell viability with FGF-2 treatment (**Fig. 2c**). Based on our results of the dose dependent assay and XTT assay, we selected the 20 ng/ml FGF-2 concentration for further experiments. Our results confirmed that FGF-2 increases bone nodule formation and decreases cell proliferation in GCT stromal cells in culture.

**Figure 2:** Bone nodule forming assay. (**a**). GCT stromal cells were induced into osteoblastic differentiation by exposure to FGF-2. Alizarin staining was used for bone nodules, and visualized by phase-contrast microscopy. (**b**). Von Kossa staining were used to determined GCT stromal cells osteoblastic differentiation by exposure to FGF-2. Bone nodules are visualized by phase-contrast microscopy. (**c**). **XTT assay.** A decreased number of mitochondrial active cells were seen in FGF-2 treated cells when compared to untreated GCT stromal cells. GCT untreated cells were used as a control (CT).

### FGF-2 promotes osteogenic marker expression in GCT stromal cells

We next determined the effect of FGF-2 on the molecular expression of markers for osteogenic differentiation in GCT stromal cells. Cells were treated with 20 ng/ml FGF-2 supplemented media. As shown in Figure **3a**, FGF-2 increased osteopontin (an early osteoblastic marker), osteocalcin (a late osteoblastic marker) and alkaline phosphatase (mature osteoblast marker) mRNA and protein expression *in vitro* and verified by quantification analysis (**Fig. 3b**). In immunofluorescence microscopy, we also observed an increase of cell-cell attachment, which is required for bone nodule formation (**Fig. 3c**). Additionally, we observed an increase in intensity of alkaline phosphatase (ALP activity) in FGF-2 treated GCT stromal cells (**Fig. 3d**).

**Figure 3:** FGF-2 promotes osteogenic differentiation in GCT cells. (**a**). qRT-PCR analysis representing an increase in osteogenic differentiating markers ALP, OPN, and OC (*p<0.05*). These results are verified at the protein level by Western blot analysis. (**b**). Quatification analysis showing an increasing OPN protein level in all FGF2 treated cell types when compared to untreated cells. (**c**). Subcellular localization of OPN in GCT stromal cells was detected by immunofluorescence using an anti-OPN monoclonal antibody. DAPI (blue) staining indicated the nuclei. F = FGF-2 treated cells. (**d**). GCT cells were incubated with and without FGF-2 (20 ng/mL) for 48 h. The cells were then analyzed for ALP activity. Data represent mean ±SD. *p<0.05.

### Effect of FGF-2 on transcription factors responsible for osteoblastic differentiation

To confirm that FGF-2 enhances osteogenic differentiation signaling in GCT stromal cells, the cells were treated with supplemental media containing 20 ng/ml FGF-2 and compared with untreated GCT stromal cells. Both PCR (**Fig. 4a**) and Western blot (**Fig. 4b**) data confirmed an increase in Runx2 mRNA and protein expression with FGF-2 treatment; whereas TWIST1 expression was decreased in all GCT samples (**Fig. 4a, b and c**). These results indicate that FGF-2 signaling may enhance osteoblast differentiation by suppressing TWIST1 and up regulating Runx2 in cultured GCT stromal cells.

**Figure 4:** FGF-2 stimulation effects on osteoblastic transcription factors in GCT cells. Quantitative RT-PCR, Western blot and quantification analysis representing a significant decrease in TWIST1 and a significant increase in Runx2 mRNA and protein levels in GCT cells treated with FGF-2 (GCT1F, and GCT2F,) when compared to the GCT untreated (GCT1, and GCT2) FGF-2 cells.

### TWIST1 inhibits osteogenic differentiation

To determine the role of TWIST1 in primary GCT mesenchymal stromal cell differentiation, we generated a TWIST-pcDNA 3.1 construct and transfected as described in primary GCT mesenchymal stromal cells. PCR data confirmed successful transfection and overexpression of TWIST in two GCT cell lines (**Fig. 5a**). TWIST mRNA levels were elevated >8-fold in GCT-1 and >7-fold in GCT-2 transfected cells when compared to GCT untransfected cells. We observed a decrease in FGFR-2IIIc expression in TWIST overexpressing GCT stromal cells when compared to GCT untransfected cells (**Fig. 5b**). Furthermore, we indentified a decrease in matrix mineralization with TWIST1 over-expressing cells treated with FGF-2 compared to GCT cells (**Fig. 5c**). We next determined that TWIST1 over-expression in FGF-2 stimulated GCT stromal cells suppresses ALP, OPN and OC (osteoblastic differentiation markers) at the mRNA level (**Fig. 5d**). These results reveal that TWIST1 over-expressing GCT stromal cells inhibit FGF-2 stimulated osteoblastic differentiation of GCT stromal cells, possibly by inhibiting the expression of the FGF-2 receptor, FGFR-2IIIc.

**Figure 5:** TWIST1 suppresses osteogenic differentiation. (**a**). Quantitative RT-PCR analysis representing higher TWIST1 expression in transfected GCTT1, GCTT2 cells compared to untransfected (UT) GCT stromal cells. (**b**). Quantitative PCR analysis showing a 60% decrease of FGFR2-IIIc expression in GCTT1 and a 50% decrease of FGFR2-IIIc expression in GCTT2 stromal cells (*p<0.05). (**c**). GCT cells were transfected with TWIST1 and matrix mineralization compared to control (CT) and FGF-2 treated GCT cells. (**d**). TWIST1 over-expression showed a significant decrease in ALP, OPN and OC mRNA levels in GCT cells treated with FGF-2 (GCTT1, and GCTT2,) when compared to the GCT untreated (UT) FGF-2 cells.

### FGFR2 knockdown and osteoblastic differentiation in GCT cells

To determine that FGF-2 ligand enhances osteoblast differentiation and osteogenic capacity in cultured GCT stromal cells through FGFR-2IIIc signaling, FGFR-2IIIc expression was knocked down by transient transfection of siRNA in GCT stromal cells. We depleted FGFR-2IIIc expression in the mesenchymal stromal cells of GCT in two representative primary cell lines and subsequently measured the expression level of TWIST1, Runx2, and ALP mRNA. We successfully obtained approximately 70% FGFR2-IIIc mRNA knock down in both primary cell lines (**Fig. 6a**). Knock down of FGFR2-IIIc resulted in approximately a 1.5 fold increase in TWIST1 expression and a significant decrease in Runx2 and ALP expression (**Fig. 6b** **,** ***p*** **<0.01**).

**Figure 6:** The effect of FGFR-2IIIc siRNA on mRNA expression in the GCT stromal cells. (**a**). FGFR2 siRNA transfection resulted in a 70% decrease in FGFR-2IIIc expression in GCT stromal cells. (**b**). Quantitative RT-PCR was used to represent the expression of ALP, Runx2 and TWIST following FGFR-2IIIc knockdown (KO) in GCT cells. Results are the average of three replicate experiments. FGFR-2IIIc knockdown resulted a 1.5 fold increase of TWIST1 expression and a significant decrease in Runx2 and ALP expression *(p<0.05).*

### FGFR-2IIIc mediates osteoblast differentiation in GCT cells through ERK1/2 signaling

ERK1/2 is one of the main downstream targets of activated FGFRs. In order to determine whether the ERK1/2 signaling pathway plays a role in osteoblastic differentiation in GCT stromal cells, we investigated changes in ERK1/2 signaling with increased expression of FGFR2-IIIc. We found that FGF-2 stimulation was associated with an increase in phosphorylated ERK1/2 expression (**Fig. 7a and b**). After confirming that phosphorylated ERK1/2 expression is stimulated by FGF-2 in GCT stromal cells, next we evaluated the effects of ERK inhibitor on the expression of TWIST1 and osteoblastic differentiation markers at the mRNA level. Treatment of GCT mesenchymal stromal cells from two representative primary GCT cell lines with the ERK-inhibitor PD98059 under FGF-2 stimulation resulted in a significant reduction of ALP, OPN and OC mRNA levels, with optimized 1 nM concentration of inhibitor (**Fig. 7c**).We also observed a slight increase in TWIST1 expression in both cell lines. Our results suggest that FGFR2 signaling plays an essential role in osteoblastic differentiation in GCT stromal cells, possibly via ERK signaling.

**Figure 7:** FGF2 signaling through ERK in osteoblast differentiation in GCT stromal cells. (**a**) Western blot analysis (**b**) and quantification showed that FGF-2 stimulation resulted in increased phosphorylation of ERK1/2 (p-ERK1/2), compared to untreated GCT cells. β-Actin was used as loading control. (**c**). Inhibition of osteoblastic gene expression by ERK inhibitor in GCT stromal cells based on real-time RT-PCR. GCT stromal cells were treated with 1 nM ERK-inhibitor PD98059 (all diluted in DMSO) for 24 h in serum-free medium. mRNAs were purified, cDNAs were synthesized, and the samples were analyzed by real-time PCR. The ΔΔCT method was used to calculate the real-time RT-PCR fold change using RPS18 mRNA as an endogenous control, and all changes in expression are relative to the control without treatment. Three independent real-time PCR runs were performed on each sample.

## Discussion

GCT is characterized by the presence of osteoclast-like giant cells, a mononuclear component, and mesenchymal stromal cells. To date, the oncogenesis of GCT remains unknown as the neoplastic cells appear to be preosteoblastic cells that do not undergo terminal osteoblastic differentiation [2], [3], [6]. Mesenchymal stromal cells are able to differentiate into mature osteoblasts under appropriate stimulation with FGFs or other proteins [11]. However, the mechanisms by which these factors control osteogenesis have not been fully elucidated. In this study, we have identified a regulatory pathway involving FGF-2 and FGFR2-IIIc, which plays a role in osteogenic differentiation in GCT stromal cells.

FGFR2 signaling plays an essential role in skeletal development in mouse and human genetics [11]. Several FGFR expression profile studies indicated that FGFR1 and FGFR2 are the main receptors expressed in osteoblasts whereas FGFR3 is the most important growth factor for chondrocytes [11], [31]. However, the expression of specific FGFRs and their role in GCT stromal cell differentiation remains unknown. Several microarray and proteomics studies were conducted using giant cell tumor of bone and FGFR2 and FGF ligands were observed *in vivo* [32]. We observed very high expression of FGFR2-IIIc, but not FGFR2-IIIb, in GCT stromal cells when compared to human fetal osteoblastic (hFOB) 1.19 cells, suggesting that FGFR2-IIIc plays a prominent role in these cells. Higher expression of FGFR2-IIIc in GCT stromal cells could be an important transducer of FGF signals in osteoblastic differentiation. We also observed an increase in the expression of FGFR2-IIIc in response to FGF-2 ligand in a dose dependent manner.

To determine a more precise role for FGFR2-IIIc in GCT stromal cell differentiation, cells were treated with FGF-2 and it was observed that FGF-2 promotes cell differentiation in GCT stromal cells. FGF-2 treated cells actively promoted matrix mineralization when compared to untreated GCT cells. Although others have found FGF-2 signaling to enhance cell proliferation in bone cells [9], [33], the specific function of FGF-2 in cell proliferation in bone tumor cells is poorly understood. To investigate this important concept, an XTT assay was performed and we observed that FGF-2 decreased GCT stromal cell proliferation. Cells treated with FGF-2 have a significant decrease in their growth rate, which may be due to an increase in differentiation. In general, upon differentiation of various tissues and cell lines from different organisms, proliferation is uniformly suppressed [34], [35].

Based on these findings, we sought to determine whether FGF-2 would functionally promote osteoblastic differentiation signaling in GCT stromal cells. Quantitative RT-PCR analysis showed that FGF-2 induced an approximately 2-fold increase in mRNA expression of Runx2 at 48h in culture. Runx2 is one of the earliest and most specific markers of osteoblast differentiation, capable of inducing differentiation by regulating expression of numerous osteoblast-specific genes [20]. Runx2 interacts with multiple co-regulating transcription factors and signaling proteins, forming multimeric complexes. These complexes then either transactivate or repress target genes during osteogenic differentiation [36]–[38]. Thus, Runx2 is a transcription factor that plays the role of the initial and terminal “switch” responsible for osteoblastic cell differentiation. Osteopontin and ALP mRNA expression levels also increased in GCT cells after treating with FGF-2 when compared to the untreated GCT stromal cells, whereas TWIST1 mRNA expression was decreased. These findings are not surprising given that in a mouse model where the TWIST1 gene was overexpressed, Runx2 expression was undetectable during development [19], [26]. Additionally, TWIST1 has been shown to have negative involvement in osteoblastic differentiation by interfering with Runx2 function at early stages of osteogenesis [39].

Furthermore, to confirm that FGFR2-IIIc signaling is involved in osteoblastic differentiation, FGFR2-IIIc expression was knocked down in the GCT cells using siRNA. A yield of 70% FGFR2-IIIc knock down resulted in an approximately 1.5 fold increase in TWIST1 expression and a significant decrease in RunX2 and ALP mRNA expression in GCT stromal cells when compared to the untreated cells. Over-expression of TWIST1 expression in GCT stromal cells inhibits GCT cell differentiation and matrix mineralization. Altogether, our data supports a definite role for FGFR2-IIIc signaling in osteoblastic differentiation of GCT stromal cells *in vitro*.

Several studies identified that the ERK1/2 signaling may be important in osteogenic differentiation [40]–[42]. ERK1/2 is one of the main downstream targets of activated FGFRs [12], [43]. Our data indicates that FGF-2 treatment of GCT cells resulted in activation of ERK1/2 in these cells. Our findings indicate that the increasing levels of FGF-2 are functionally correlated with FGFR2-IIIc which activates downstream ERK1/2 signaling pathways of osteoblast differentiation in GCT stromal cells. Inhibitors of ERK1/2 PD98059 abolished the increased osteoblast gene expression at the mRNA level. The FGF-2 induced osteoblastic differentiation gene expression was strongly suppressed by the ERK inhibitor. Our results suggest that FGFR2-IIIc and ERK1/2 pathways mediate, at least in part, the positive effect of FGF-2 stimulation on osteoblast differentiation in GCT stromal cells. These signaling pathways may therefore serve as targets in treatment strategies for this destructive tumor and other diseases of the musculoskeletal system.

In summary, our data indicates that FGFR2-IIIc signaling enhances the osteogenic differentiation program in GCT stromal cells. *In vitro* experiments revealed that this effect results from mechanisms involving up regulation of Runx2 and down regulation of TWIST1 (**see proposed signaling mechanism** **Fig. 8**). The increasing levels of FGFR2-IIIc are functionally correlated with the differentiation process in GCT stromal cells and therefore the targeting of the FGFR2-IIIc pathway may serve as a useful tool for differentiation therapy in GCT patients.

**Figure 8:** Proposed signaling mechanisms representating the osteogenic differentiation model induced by FGF-2 in GCT stromal cells. FGFR2-IIIc is activated by FGF-2, which in turn increases ERK1/2 signaling in GCT stromal cells. ERK1/2 activates Rux2 expression and suppresses TWIST1 expression, thus stimulating osteoblastic differentiation.
